# Effects of CIK Cell Therapy Combined with Camrelizumab on the Quality of Life in Patients with Nasopharyngeal Carcinoma and Analysis of Prognostic Factors

**DOI:** 10.1155/2022/5655009

**Published:** 2022-05-09

**Authors:** Tao Feng, Xiu Luo, Wenping Cao, Rongjun Man, Xinrong Feng, Yujie Song

**Affiliations:** Department of Otolaryngology, Zibo Central Hospital, Zibo 255000, Shandong, China

## Abstract

**Objective:**

To investigate the effects of CIK (cytokine-induced killer) cell therapy combined with camrelizumab on the quality of life in patients with nasopharyngeal carcinoma and prognostic factors.

**Methods:**

In this retrospective study, the materials of 80 patients with nasopharyngeal carcinoma treated in our hospital (February 2017–February 2019) were retrospectively analyzed, and they were equalized into experimental group (*n* = 40) and control group (*n* = 40) according to the order of admission. Both groups received 200 mg of camrelizumab on day 1 combined with 10 mg of anrotinib from day 2 to day 4. The patients received the above program every 3 weeks and 4 treatment cycles. The experimental group also received CIK cell therapy simultaneously. The patients' quality of life, immune indexes, local control, metastasis, and survival rate were compared between the two groups, and the prognostic factors were analyzed by logistic analysis.

**Results:**

Compared with the control group, the experimental group achieved much higher scores of physical well-being (18.38 ± 2.31), social/family well-being (16.40 ± 2.24), emotional well-being (15.35 ± 2.30), functional well-being (17.30 ± 2.20), and head and neck cancer subscale (15.40 ± 2.01, *P* < 0.001) and eminently better immune indexes (*P* < 0.001) after treatment. During the 24-month follow-up, there were 2 recurrent cases (5.0%) and 2 cases (5.0%) with distant metastasis among the 40 patients in the experimental group; there were 8 recurrent cases (20.0%) and 7 cases (17.5%) with distant metastasis among the 40 patients in the control group. In the experimental group, the median survival period was 18 months and the 2-year survival rate was 97.5% (39/40). In the control group, the median survival period was 14 months and the 2-year survival rate was 85.0% (34/40). Among the 80 patients, 7 cases (8.75%) died and 73 cases (91.25%) survived. After conducting the single-factor analysis, remarkable differences in the cases of IV stage, quality of life after treatment, and immune indexes after treatment between the survival group and the death group were observed (*P* < 0.05). According to the multiple-factor analysis, the clinical stage and immune indexes were identified as the prognostic factors.

**Conclusion:**

CIK cell therapy combined with camrelizumab can enhance the life quality and immune function of the patients with nasopharyngeal carcinoma, thus improving their prognoses.

## 1. Introduction

Nasopharyngeal carcinoma, as a malignant tumor originating from the epithelium of the nasopharyngeal mucosa, mostly presents in the hanging wall and sidewall of the nasopharynx. Its incidence is 30/100,000–50/100,000, and it is most prevalent among the yellow race [1, 2]. Therefore, deeper research on this disease can reduce the medical burden in China. The current academic community believes that nasopharyngeal carcinoma is closely related to Epstein–Barr virus infections, genetic and environmental factors, and poor dietary habits [3]. The patients with nasopharyngeal carcinoma do not show specific symptoms in the early stage, but develop tinnitus, hearing decrease, headache, diplopia, cranial nerve palsy, and other symptoms with disease progression [4, 5], which indicates that the patients are mostly in the middle and late stages of the disease and their quality of life is unsatisfactory [6]. Radiotherapy, chemotherapy, targeted therapy, and surgery are all important approaches to treating nasopharyngeal carcinoma, among which radiotherapy, chemotherapy, and surgery are conventional treatments, while targeted therapy is a more cutting-edge treatment. The targeted therapy can specifically block the signaling pathways which affect the growth of tumor cells, thus preventing the proliferation of tumor cells and treating the disease. In addition to targeted therapy, immunotherapy is also a cutting-edge therapeutic measure. In recent years, the immunotherapy dominated by PD-1/PD-L1 immune checkpoint inhibitors has been gradually applied to the comprehensive treatment regimen for various types of tumors. Camrelizumab is the third PD-1 drug made in China after toripalimab and sintilimab and can activate T cells by blocking PD-1/PD-L1 binding, thereby weakening the immunosuppression within the patients' organism and enhancing the tumor-killing effect [7, 8]. Zhou et al. gave the patients with advanced nasopharyngeal carcinoma targeted therapy combined with immunotherapy (anrotinib + camrelizumab), and the patients' recheck showed that they had shrunken lesions, significantly relieved cough and active shortness of breath, and remarkably improved quality of life [9], suggesting that anrotinib + camrelizumab has treatment effect on the patients with nasopharyngeal carcinoma.

Camrelizumab has satisfactory effects on treating nasopharyngeal carcinoma because the immune function of patients with nasopharyngeal carcinoma decreases with the growth of the tumor. The specific and nonspecific cells and humoral immune function of the patients with advanced nasopharyngeal carcinoma are inhibited, and camrelizumab can enhance their immune function. With the further development of tumor immunology, the treatment methods for making up the immunodeficiency are gradually increasing, and CIK (cytokine-induced killer) cell therapy is one of the treatment methods. CIK cell, as one of the immunocompetent cells, has the antitumor activity of T lymphocytes, and it can enhance the patients' treatment effects with fast cell proliferation and strong antitumor activity [10]. Some current literature has explored the effects of CIK cells on treating nasopharyngeal carcinoma, but no study investigates the combination of CIK cells and camrelizumab. Therefore, it is unclear in the academic community whether the combination can more effectively enhance the immune indexes of the patients and improve their prognoses. This study selected 80 patients with nasopharyngeal carcinoma as the research objects, aiming to investigate the effects of CIK cell therapy combined with camrelizumab on the quality of life in patients with nasopharyngeal carcinoma and the prognostic factors.

## 2. Materials and Methods

### 2.1. Research Design

This was a retrospective study. This study was conducted in our hospital from February 2017 to February 2019, aiming to investigate the effects of CIK cell therapy combined with camrelizumab on the quality of life in patients with nasopharyngeal carcinoma and prognostic factors. This study adopted the double-blind method, and both the research objects and researchers did not know the grouping in this study. The research designers were responsible for arranging and controlling all the trials.

### 2.2. General Data

The materials of 80 patients with nasopharyngeal carcinoma who were treated in our hospital (February 2017–February 2019) were retrospectively analyzed, and all the patients were diagnosed as the cases with nasopharyngeal carcinoma after the histological or cytological examination [11]. The patients were treated in our hospital in the whole course, and their survival time is expected to last more than 3 months. All the patients in this study did not have hearing impairment, speech disorder, unconsciousness, or mental illness, and they could normally communicate with other people and coordinate the follow-up. The following patients were excluded from this study: (1) the patients were complicated with infectious diseases, systemic diseases, or secondary tumors; (2) the patients had renal or liver dysfunction; (3) the patients' blood system was abnormal; (4) the patients' electrocardiogram was abnormal; (5) the patients were under 18 years old; (6) the patients were lost during follow-up; (7) the patients' Karnofsky performance status (KPS) scores were lower than 60 points; (8) the patients were pregnant or lactating; (9) the patients had the history of mental illness or malignant tumor.

The 80 patients were equalized into experimental group (*n* = 40) and control group (*n* = 40) according to the order of admission. The pathological type of all the patients was squamous cell carcinoma. In the experimental group, there were 29 males and 11 females, with the average age of (50.35 ± 5.25) years. In terms of the clinical stage, there were 2 cases in stage I, 12 cases in stage II, 20 cases in stage III, and 6 cases in stage IV. In the control group, there were 30 males and 10 females, with the average age of (50.30 ± 5.19) years. In terms of the clinical stage, there were 3 cases in stage I, 14 cases in stage II, 18 cases in stage III, and 5 cases in stage IV. No remarkable difference in the baseline data between the two groups was found (*P* > 0.05), and the two groups were comparable.

### 2.3. Steps

This study included 80 patients, and they were equalized into experimental group (*n* = 40) and control group (*n* = 40) according to the order of admission. On the day when the patients agreed to participate in the study, the study team collected the patients' sociodemographic and clinical data. Then, both groups received camrelizumab combined with anrotinib, and the experimental group also received CIK cell therapy at the same time. The follow-up for the patients lasted for 24 months, and the patients' quality of life, immune indexes, local control, metastasis, and survival rate were compared between the two groups, and prognostic factors were analyzed.

### 2.4. Moral Consideration

This study conformed with the principles of *Declaration of Helsinki (2013)* [12]. The patients were informed of the study purpose, significance, contents, and confidentiality and had signed the informed consent.

### 2.5. Methods

#### 2.5.1. Control Group

The control group received camrelizumab combined with anrotinib. The patients were given 200 mg of camrelizumab (Suzhou Suncadia Biopharmaceuticals Co., Ltd., NMPA Approval No. S20190027) on day 1 and received 10 mg of anrotinib (Jiangsu Chia Tai-Tianqing Pharmaceutical Co., Ltd., NMPA Approval No. H20180002) from day 2 to day 4. The patients received the above program every 3 weeks and 4 treatment cycles.

#### 2.5.2. Experimental Group

The experimental group received CIK cell therapy based on the treatment given to the control group. The blood collection machine (Suzhou Laishi Transfusion Equipment Co., Ltd., NMPA Approval No. 20173664660) was adopted to collect the patients' peripheral blood mononuclear cells. Each patient was drawn (1–4) × 10^9^ cells, with the volume of 40–70 mL. In a laboratory meeting the standard of GMP lab, the cell concentration was regulated to (1–2) × 10^6^/mL in the serum-free medium (GIBCO AIM-V). Then, the cells were put in the air-permeable culture bag and 1000 U/ml of IFN-*γ* was added in the first day. After culturing for 24 hours, 300 U/ml of IL-2 and IL-1 and 350 ng/ml of OKT were added to the bag and the cells were cultured in suspension at 37°C and in 5% of CO_2_ (Thermo Forma 311). The culture medium was changed every 4 hours, the cells were regulated to 1 × 10^6^/mL, and 300 U/ml of IL-2 was readded. Besides, 350 ng/ml of OKT was readded every 8 hours when readding IL-2. From the second week, CIK cells were collected and 1/3 of the CIK cells suspension was taken every time. After centrifuging, washing, and resuspending, 400–500 mL of CIK cells suspension was made. On the 10th, 13th, and 15th days of culturing, the CIK cells produced by induced culture were reinfused to the patients' body. Before reinfusing, the CIK cells presented negative in the bacterium, fungus, and mycoplasma tests, and the reinfused cells were above (2–6) × 10^6^.

### 2.6. Observational Criteria

1. Quality of life [13]: the patients' quality of life 1 week before and 1 week after receiving camrelizumab combined with anrotinib was evaluated. The Functional Assessment of Cancer Therapy-Head and Neck (FACT-H＆N (V4.0)): FACT-G and FACT-HN was adopted. This scale included 5 domains of physical well-being (PWB), social/family well-being (SWB), emotional well-being (EWB), functional well-being (FWB), and head and neck cancer subscale (HNS). The GP1-GP7, GE1-GE6, HN2, HN3, HN6, HN8, and HN9 were the reverse items, and the rest were forward ones. For all the items, higher scores indicated better quality of life. Relevant studies confirmed that this scale had good reliability and validity for the patients with nasopharyngeal carcinoma, and this scale could be used to assess the quality of life of the Chinese patients with nasopharyngeal carcinoma.
2. Immune indexes: the patients' immune indexes 1 week before and 1 week after receiving camrelizumab combined with anrotinib were assessed. The flow cytometry (Beckman Coulter, Inc., NMPA (I) 20173401372) was adopted to determine the patients' levels of T lymphocyte subsets (CD3^+^, CD4^+^, and CD8^+^) and to calculate Th1/Th2.
3. Local control and metastasis: three months after the end of treatment, follow-up began and lasted for 24 months. Patients were rechecked every 3 months, with a physical examination, hematology, CT examinations, ultrasonography, and fiberoptic pharyngorhinoscopy. In addition, the patients received nasopharyngeal MRI every 6 months to investigate the local recurrence or the recurrence of cervical lymph nodes. All the recurrence cases were pathologically confirmed.
4. Survival rate: the patients' 2-year survival rate in the two groups were recorded and analyzed.
5. Analysis of prognostic factors: the patients were divided into the survival group and the death group according to their survival state, and the single-factor analysis and multiple-factor analysis were adopted to investigate the prognostic factors.

### 2.7. Statistical Treatment

The professional statistical software SPSS20.0 was adopted for data processing, and GraphPad Prism 7 (GraphPad Software, San Diego, USA) was used to draw graphs of the data in this study. This study included count data and measurement data, which were tested by *X*^2^ and *t*. When *P* < 0.05, the differences were considered statistically significant.

## 3. Results

### 3.1. Comparison of the Quality of Life

Compared with the control group, the experimental group had much higher quality of life (*P* < 0.001; Figure 1).

In Figure 1, the abscissa, respectively, referred to before treatment and after treatment from left to right. The line with dots represented the experimental group, and the line with squares represented the control group.

Figure 1(a) shows PWB scores; before treatment, no statistical difference in PWB scores between the experimental group and the control group was discovered (20.90 ± 1.87 vs. 20.35 ± 2.24, *P* > 0.05); after treatment, the experimental group achieved much higher PWB score compared with the control group (18.38 ± 2.31 vs. 15.08 ± 3.30, *P* < 0.001).

Figure 1(b) refers to SWB scores; before treatment, no statistical difference in SWB scores between the experimental group and the control group was discovered (20.10 ± 1.91 vs. 20.45 ± 2.21, *P* > 0.05); after treatment, the experimental group achieved much higher SWB score compared with the control group (16.40 ± 2.24 vs. 12.75 ± 2.96, *P* < 0.001).

Figure 1(c) refers to EWB scores; before treatment, no statistical difference in EWB scores between the experimental group and the control group was discovered (19.00 ± 1.97 vs. 19.08 ± 2.36, *P* > 0.05); after treatment, the experimental group achieved much higher EWB score compared with the control group (15.35 ± 2.30 vs. 12.95 ± 2.47, *P* < 0.001).

Figure 1(d) refers to FWB scores; before treatment, no statistical difference in FWB scores between the experimental group and the control group was discovered (19.18 ± 2.00 vs. 19.38 ± 2.21, *P* > 0.05); after treatment, the experimental group achieved much higher FWB score compared with the control group (17.30 ± 2.20 vs. 12.55 ± 2.69, *P* < 0.001).

Figure 1(e) refers to HNS scores; before treatment, no statistical difference in HNS scores between the experimental group and the control group was discovered (19.15 ± 1.97 vs. 19.33 ± 2.27, *P* > 0.05); after treatment, the experimental group achieved much higher HNS score compared with the control group (15.40 ± 2.01 vs. 12.90 ± 2.54, *P* < 0.001).

### 3.2. Comparison of the Immune Indexes

Compared with the control group, the experimental group achieved eminently better immune indexes after treatment (*P* < 0.001; Figure 2).

In Figure 2, the abscissa, respectively, referred to before treatment and after treatment from left to right. The line with dots represented the experimental group, and the line with squares represented the control group.

Figure 2(a) refers to the comparison of CD3^+^; before treatment, no statistical difference in CD3^+^ between the experimental group and the control group was discovered (49.65 ± 2.12 vs. 49.67 ± 2.15, *P* > 0.05); after treatment, the experimental group achieved much higher CD3^+^ compared with the control group (64.11 ± 2.41 vs. 55.00 ± 4.45, *P* < 0.001).

Figure 2(b) refers to the comparison of CD4^+^; before treatment, no statistical difference in CD4^+^ between the experimental group and the control group was discovered (26.12 ± 2.10 vs. 26.24 ± 2.55, *P* > 0.05); after treatment, the experimental group achieved much higher CD4^+^ compared with the control group (36.24 ± 2.10 vs. 29.32 ± 3.65, *P* < 0.001).

Figure 2(c) refers to the comparison of CD8^+^; before treatment, no statistical difference in CD8^+^ between the experimental group and the control group was discovered (24.12 ± 1.20 vs. 24.15 ± 1.22, *P* > 0.05); after treatment, the experimental group achieved much higher CD8^+^ compared with the control group (27.65 ± 1.41 vs. 23.70 ± 3.88, *P* < 0.001).

Figure 2(d) refers to the comparison of Th1/Th2; before treatment, no statistical difference in Th1/Th2 between the experimental group and the control group was discovered (0.57 ± 0.05 vs. 0.59 ± 0.04, *P* > 0.05); after treatment, the experimental group achieved much higher Th1/Th2 compared with the control group (1.12 ± 0.08 vs. 0.81 ± 0.15, *P* < 0.001).

### 3.3. Comparison of the Local Control and Metastasis

The follow-up rate of the 80 patients was 100.0%, and the follow-up lasted for 24 months. Among the 40 patients in the experimental group, the recurrence occurred in 2 cases (5.0%, one with local recurrence alone and another with the recurrence of cervical lymph node alone) and distant metastasis occurred in two cases (5.0%, one taking distant metastasis as the condition of treatment failure and another suffering from distant metastasis after recurrence). Among the 40 patients in the control group, recurrence occurred in 8 cases (20.0%, three cases with local recurrence alone, three cases with the recurrence of cervical lymph node alone, and two cases with local recurrence and cervical recurrence simultaneously) and distant metastasis occurred in 7 cases (17.5%, 4 cases taking distant metastasis as the condition of treatment failure and 3 cases suffering from distant metastasis after recurrence).

### 3.4. Comparison of the Survival Rate

In the experimental group, the median survival period was 18 months and the 2-year survival rate was 97.5% (39/40). In the control group, the median survival period was 14 months and the 2-year survival rate was 85.0% (34/40). Remarkable difference in the survival rates between the two groups was observed (*P* < 0.05; Figure 3).

### 3.5. Analysis of the Prognostic Factors

After conducting single-factor analysis, remarkable differences in the cases of IV stage, quality of life after treatment, and immune indexes after treatment between the survival group and the death group were observed (*P* < 0.05). According to the multiple-factor analysis, the clinical stage and immune indexes were identified as the prognostic factors (Tables 1 and 2).

## 4. Discussion

Nasopharyngeal carcinoma is a common malignant tumor occurring in the head and neck, and its pathological type is mostly squamous cell carcinoma [14]. The patients with nasopharyngeal carcinoma do not have specific symptoms in the early stage. Therefore, when the patients are diagnosed as the cases with nasopharyngeal carcinoma, they are often in the middle or late stage with the 5-year survival rate of under 15.0%, and 70.0% of them have metastasis [15]. The general survival status of the patients is not optimistic. Currently, radiotherapy and chemotherapy, as the main treatment methods for nasopharyngeal carcinoma, have unsatisfactory treatment effect for the patients in the middle or late stage and do not significantly improve the patients' 5-year survival rate, and their quality of life is poor in general [16, 17]. With the development of tumor immunology, the academia has gradually clarified that tumor immune escape is one of the key mechanisms of the occurrence and development of malignant tumors [18]. The onset of nasopharyngeal carcinoma is closely related to Epstein–Barr virus (EBV). EBV, a member of the lymphotropic virus genus in Herpesviridae, has the biological characteristics of specifically infecting human B cells *in vitro* and *in vivo*. The tumor tissues release a large amount of immunosuppressive factors during growth to inhibit T lymphocytes from differentiating and being mature and to induce T cells from differentiating to suppressor T cells. As a result, the percentage of T cell subsets is decreased and specific cytotoxic T lymphocytes conducive to killing EB virus are absent, leading to the treatment failure finally [19, 20]. Therefore, improving the patients' immune function is the emphasis of treating nasopharyngeal carcinoma in clinic. Camrelizumab, a common drug for immunotherapy of nasopharyngeal carcinoma, is a humanized monoclonal antibody and effectively blocks the binding of PD-1/PD-L1, which plays a key role in tumor immune escape. Besides, camrelizumab inhibits tumor growth by activating T cells to produce sustained antitumor effect. In phase I trials of evaluating the application of single carrilizumab and the combination of carrilizumab with gemcitabine and cisplatin, the carrilizumab has been found to have good activity in patients with recurrent or metastatic nasopharyngeal carcinoma [21]. For patients who have received first-line treatment, the single carrilizumab can still prolong their progression-free survival and improve the complete remission rate, indicating the value of carrilizumab in treating the nasopharyngeal carcinoma. It is worth mentioning that carrilizumab can improve the efficacy of the patients whose immunosuppression is aggravated by radiotherapy and chemotherapy [22]. In this study, the patients' immune levels were enhanced in both groups after treatment, confirming the definite effect of carrilizumab on improving the patients' immune function.

The application of kareolizumab means that immunotherapy for nasopharyngeal carcinoma has entered a new era, and the progresses in molecular biology and bioengineering technology have enabled the immunotherapy methods to gradually increase. CIK is a new type of immunocompetent cell that can be used for nasopharyngeal carcinoma treatment [23]. CIK cells are the T cells obtained by cultivating human peripheral blood mononuclear cells with various cytokines and are characterized with broad tumoricidal spectrum and high efficiency in killing tumors. The tumoricidal activity of CIK cells is much higher than that of lymphokine-activated killer cells and cytotoxic T cells [24]. Therefore, CIK cells are receiving increasing attention in clinic. Many studies have confirmed that CIK cells can enhance the patients' immune function, so the experimental group achieved eminently better immune indexes after treatment compared with the control group (*P* < 0.001). In addition, the recurrence and metastasis rates in the experimental group were lower than those in the control group, indicating that CIK cells exerted a potent tumor-killing effect. The cytotoxicity of CIK cells is nonspecific, and CIK cells work by binding relevant antigens to intercellular adhesion molecule-1 on the surface of target cells. In this way, CIK cells release perforins, cytolysins, and other substances which can cause the osmotic lysis of target cells. As a result, the target cells are killed. According to the study of scholars Blanchard Pierre et al., CIK cells enhance the cytotoxic effect of other immune cells by secreting a variety of cytokines, which further heightens the tumor-killing ability of CIK cells [25]. CIK cells enhance the immune function and consolidate the efficacy of other treatment measures by effectively killing tumor cells. Therefore, the experimental group had a higher survival rate and a more satisfactory quality of life.

After analyzing relevant factors, it was found that the clinical stage and immune indexes had an impact on the patients' survival rate. The impact of clinical stage on the patients' prognoses has been confirmed, and the relationship between the patients' immune function and prognoses has been demonstrated above. The results of multiple-factor analysis showed that CIK cell therapy combined with camrelizumab not only has good short-term effect but also optimizes the long-term effect by affecting the immune function, which is significant for improving the patients' prognoses. It is worth noting that the two treatment methods were performed simultaneously in this study, and if CIK cell therapy is combined with radiotherapy and chemotherapy, the CIK cell therapy should be postponed for 2 weeks to ensure the patients' recovery.

In conclusion, CIK cell therapy combined with camrelizumab can enhance the life quality and immune function of the patients with nasopharyngeal carcinoma, thus improving their prognoses and reducing the medical burden of such patients in China.

## Figures and Tables

**Figure 1:** Comparison of the quality of life ($\bar{x}$*x* ± *s*, points).

**Figure 2:** Comparison of the immune indexes ($\bar{x}$ ± *s*).

**Figure 3:** Comparison of the survival rate. Note: the full line represents the control group, and the dashed line represents the experimental group.

**Table 1:** Single-factor analysis of the patients' prognoses.

Group	Survival group (*n* = 73)	Death group (*n* = 7)	*X* ^2^/*t*	*P*
*Sex*			0.021	0.884
Male	54	5		
Female	19	2		
Age (years old)	50.29 ± 5.13	50.71 ± 6.04	0.204	0.839

*Clinical stages*				
I stage	5	0	0.511	0.475
II stage	26	0	3.694	0.055
III stage	37	1	3.394	0.065
IV stage	5	6	33.499	<0.001

*FACT-H&N scores after treatment*				
PWB	17.37 ± 2.51	10.00 ± 2.98	7.307	<0.001
SWB	15.08 ± 2.64	9.29 ± 3.69	5.350	<0.001
EWB	14.52 ± 2.43	10.29 ± 1.91	4.466	<0.001
FWB	15.38 ± 2.97	10.14 ± 4.09	4.313	<0.001
HNS	14.56 ± 2.20	9.86 ± 2.64	5.310	<0.001

*Immune indexes after treatment*				
CD3+	60.69 ± 4.46	47.76 ± 4.86	7.275	<0.001
CD4+	33.63 ± 3.57	23.88 ± 4.33	6.781	<0.001
CD8+	26.52 ± 1.98	16.83 ± 3.90	11.191	<0.001
Th1/Th2	1.00 ± 0.15	0.59 ± 0.19	6.753	<0.001

**Table 2:** Multiple-factor analysis of the patients' prognoses.

Factors	*B*	Wald	*P*	OR (95% CI)
IV stage	0.235	12.140	0.001	2.351 (1.341–4.152)
PWB	−0.423	50.124	0.231	0.362 (0.637–3.576)
SWB	−0.424	51.658	0.224	0.365 (0.485–3.562)
EWB	−0.452	50.985	0.214	0.341 (1.374–3.745)
FWB	−0.458	51.214	0.234	0.232 (1.387–3.745)
HNS	−0.247	15.352	0.001	2.321 (1.558–5.658)
CD3+	−0.234	15.224	0.002	2.235 (1.568–4.972)
CD4+	−0.247	12.125	0.035	2.321 (1.487–3.241)
CD8+	−0.214	12.351	0.038	2.354 (1.569–3.984)
Th1/Th2	−0.245	11.354	0.042	2.412 (1.254–3.745)

## Data Availability

The data used to support the findings of this study are available on reasonable request to the corresponding author.
